# Lack of mitochondrial ferritin aggravated neurological deficits via enhancing oxidative stress in a traumatic brain injury murine model

**DOI:** 10.1042/BSR20170942

**Published:** 2017-11-06

**Authors:** Ligang Wang, Libo Wang, Zhibo Dai, Pei Wu, Huaizhang Shi, Shiguang Zhao

**Affiliations:** 1 Department of Neurosurgery, 1st Affiliated Hospital, Harbin Medical University, Harbin 150001, China; 2 Department of Medicine and Management, Mudanjiang Chinese Traditional Medicine Hospital, Mudanjiang 157000, China

**Keywords:** antioxidant, mitochondrial ferritin, neurological deficits, oxidative stress, traumatic brain injury

## Abstract

Oxidative stress has been strongly implicated in the pathogenesis of traumatic brain injury (TBI). Mitochondrial ferritin (Ftmt) is reported to be closely related to oxidative stress. However, whether Ftmt is involved in TBI-induced oxidative stress and neurological deficits remains unknown. In the present study, the controlled cortical impact model was established in wild-type and Ftmt knockout mice as a TBI model. The Ftmt expression, oxidative stress, neurological deficits, and brain injury were measured. We found that Ftmt expression was gradually decreased from 3 to 14 days post-TBI, while oxidative stress was gradually increased, as evidenced by reduced GSH and superoxide dismutase levels and elevated malondialdehyde and nitric oxide levels. Interestingly, the extent of reduced Ftmt expression in the brain was linearly correlated with oxidative stress. Knockout of Ftmt significantly exacerbated TBI-induced oxidative stress, intracerebral hemorrhage, brain infarction, edema, neurological severity score, memory impairment, and neurological deficits. However, all these effects in Ftmt knockout mice were markedly mitigated by pharmacological inhibition of oxidative stress using an antioxidant, N-acetylcysteine. Taken together, these results reveal an important correlation between Ftmt and oxidative stress after TBI. Ftmt deficiency aggravates TBI-induced brain injuries and neurological deficits, which at least partially through increasing oxidative stress levels. Our data suggest that Ftmt may be a promising molecular target for the treatment of TBI.

## Introduction

Traumatic brain injury (TBI) is a leading cause of death and disability, affecting more than 10 million people annually throughout the world [1,2]. TBI is commonly caused by traffic accidents, sports injuries, violent injuries, and occupational accidents, resulting in disruption of vessels, neurons and axons, and impairment in thinking, learning, language, and behavior [1,3]. Pathogenesis of TBI is usually divided into two phases: primary and secondary injuries [3]. It is generally accepted that the damage from the primary injury cannot be changed, but secondary injury can be alleviated by effective therapy [3,4]. Moreover, the secondary injury can further exacerbate the primary direct injury [5,6]. Thus, numerous studies have focused on the secondary injury.

Increasing evidence demonstrate that oxidative stress induced by aberrant accumulation of reactive oxygen species (ROS) plays an important role in the pathogenesis of TBI [6–8]. Excessive levels of oxidative stress can cause protein, nucleic acids and lipids damage, leading to neurological dysfunction [8,9]. On the contrary, the endogenous antioxidant defense system, such as GSH and superoxide dismutase (SOD), protects brain tissue from oxidative injury [10]. Following TBI, the balance between the oxidative stress and antioxidant defense system is disrupted, concomitantly with increased malondialdehyde (MDA) and nitric oxide (NO) levels and reduced GSH and SOD levels [6,7]. Importantly, this imbalance directly results in inflammation, excitotoxicity and brain edema, which further aggravates the secondary brain injury and even increases the death rate if not effectively inhibited or treated [4,6,8].

Mitochondrial ferritin (Ftmt) is a type of ferritin that accumulates specifically in the mitochondria and shares 70% homology with heavy chain of ferritin (H-ferritin) [11,12]. Nevertheless, Ftmt possesses different characteristics compared with H-ferritin. For instance, H-ferritin has an iron-responsive element (IRE), while Ftmt transcript lacks this element [11,13]. H-ferritin is widely distributed in tissues, but Ftmt is physiologically expressed mainly in the kidney, testis, brain, heart, and tissues with high oxygen consumption activity [13,14]. The tissue distribution of Ftmt exerts a protective effect in mitochondria against iron-dependent oxidative stress, indicating the involvement of Ftmt in the regulation of oxidative stress [15]. However, its exact role in oxidative stress in the pathogenesis of TBI remains poorly understood. In the present study, we observed decreased Ftmt protein expression in TBI mice brain, which correlated with increased oxidative stress levels. Ftmt deficiency greatly enhanced TBI-induced oxidative stress and neurological deficits, suggesting that Ftmt may be a novel target for the treatment of TBI.

## Materials and methods

### Animals

Male wild-type C57BL/6 mice and male Ftmt knockout mice were obtained from the Jackson Laboratory (CA, U.S.A.). Mice were housed in cages under conditions controlled for temperature (22°C) and humidity (40%), using a 12-h light/dark cycle. They had a standard rodent diet and water *ad libitum*. All the procedures were carried out in accordance with the institutional guidelines for the Care and Use of Laboratory Animals of Harbin Medical University. The protocol was approved by the Institutional Animal Care and Use Committee of Harbin Medical University. All the surgeries were performed under isoflurane anesthesia.

### Induction of TBI

The controlled cortical impact model was used to stimulate TBI *in vivo* as previously described [16]. In brief, mice were anesthetized with 3% isoflurane in 67% N_2_O/30% O_2_, and then were placed on a CMA 450 temperature controller (Harvard Apparatus, MA, U.S.A.) to maintain body temperature at +37°C. The heads of mice were fixed in a stereotactic frame of a contusion device TBI-0310 (Precision Systems and Instrumentation, Fair-124 fax, VA, U.S.A.). The skull was drilled open 1 mm away from the midline and in the middle of the bregma and lambda to create a 4 mm diameter craniotomy over the right parietal cortex. The injury was produced by a rounded metal tip (3 mm diameter), which was adjusted at an angle parallel to the surface of impact site. The impact velocity was 5 m/s, and the impact time was set as 100 ms. A deformation depth 2 mm below the dura was used. The sham mice were received same procedure without cortical impact. All mice (*n*=400) were randomly divided into eight groups: wild-type control (with no intervention) (WT control, *n*=20), knockout control (KO control, *n*=20), WT sham (*n*=20), KO sham (*n*=20), WT TBI (*n*=80), KO TBI (*n*=80), WT TBI with N-acetylcysteine (NAC) injection (WT TBI + NAC, *n*=80), and KO TBI with NAC injection (KO TBI + NAC, *n*=80). NAC was injected intraperitoneally at a dose of 5 mg/kg right after TBI surgery, and then continuously dosed once a day for 14 days. According to time points (1, 3, 7, and 14 days), the latter four groups were further divided into four subgroups (*n* = 20/group). Within WT control, WT sham and WT TBI (14-day experimental period) groups, six mice from each group were used to measure the Ftmt protein expression, oxidative stress level and immunohistochemistry, four mice were used for brain infarct volume measurement, and ten mice were used to examine the brain water content. Post-TBI, mice were monitored daily and survived to 14 days.

### Western blotting

The protein expression of Ftmt was analyzed by Western blotting as previously described [17,18]. Briefly, the brain cortex protein from injured area was extracted using RIPA buffer (Beyotime, Jiangsu, China) containing 1% protease inhibitor cocktail (Roche, Mannheim, Germany). The protein concentration was determined by Protein Assay Kit (Thermo, MA, U.S.A.). Equal protein of each sample was separated on 8% Tris/HCl polyacrylamide gel, and then transferred to a polyvinylidene difluoride membrane (Millipore, MA, U.S.A.). After blocking in 5% nonfat milk for 1 h, the membranes were incubated with primary antibodies against Ftmt (1:500; Sigma, SAB2700108, MO, U.S.A.) and GAPDH (1:1000; Santa Cruz, sc-25788, CA, U.S.A.) at 4°C overnight. At the end of incubation period, membranes were then incubated with secondary antibody (1:1000; goat anti-rabbit, Millipore, AP307P) conjugated to horseradish peroxidase (HRP) for 1 h at room temperature. Bands were visualized using an enhanced chemiluminescence system (Pierce Biotech, IL, U.S.A.). The images were captured by the gel imager (GelDox XR+, Bio-Rad, CA, U.S.A.) and the densitometry of each band was quantified by Image-pro software (Media Cybernetics, MD, U.S.A.).

### Oxidative stress evaluation

Brain cortex from injured area was extracted and homogenized in physiological saline. The homogenate was centrifuged at 4000 ***g*** for 20 min. The supernatant was collected for oxidative stress analysis, and an aliquot was used for the determination of protein concentration. GSH, an important antioxidant preventing ROS-induced cellular damage, was assessed using a kit from the Nanjing Jiancheng Bioengineering Institute (Nanjing, China). SOD, which catalyzes the dismutation of superoxide into oxygen and hydrogen peroxide, was determined according to the xanthine–xanthine oxidase system using a commercial kit (Beyotime). MDA, a marker of lipid peroxidation, was evaluated by the method of thiobarbituric acid using an MDA Assay Kit purchased from Beyotime. The level of NO was estimated using an NO Detection Kit (Cayman Chemical Company, MI, U.S.A.). The measurement of these indicators of oxidative stress was performed according to the manufacturer’s instructions respectively.

### Immunohistochemistry

Hemorrhage severity in brain isolated on days 1, 3, and 7 post-TBI was assessed using IgG immunohistochemical staining. Brain tissues were fixed in 4% buffered paraformaldehyde, embedded in paraffin, and 2-µm slides were collected. After rehydrating with a serial concentration gradient of alcohols, slides were incubated with 0.3% hydrogen peroxide to block endogenous peroxidase activity, and then incubated with mouse IgG antibody (Santa Cruz, sc-2762) in 1% bovine serum albumin (Sigma) overnight at 4°C. After incubation, slides were incubated with biotinylated secondary antibody (Zhongshan Jinqiao Bio-Technology Co. Ltd., Beijing, China), and visualized with the streptavidin-peroxidase reaction using 3,3′-diaminobenzidine. The slides were dehydrated and examined under a light microscope (magnification, ×400) (IX70, Olympus, Tokyo, Japan). The optical density (OD) values for mouse IgG staining were obtained using the “Intensity Calibration” function of Image-pro software and background OD was subtracted.

### Brain infarction volume measurement

On day 14 post-TBI, the brains were removed for infract volume measurement using the 2,3,5-triphenyltetrazolium chloride (TTC, Sigma) staining. The brain slides were stained in 2% TTC for 30 min at 37°C, and then fixed with 10% formaldehyde neutral buffer solution overnight. The infract tissues were unstained, while the red regions represented as the normal area. The size of the infarct volume was measured using the “Count/Size” function of Image-pro software, and calculated as (infarct volume/contralateral hemisphere area) × 100%.

### Brain water content

On day 14 post-TBI, the brains were removed and immediately weighed to determine wet weight using an electronic balance (BSAl24SCW, Sartorius Scientific instrument, Beijing, China). Then, the brains were dried in an oven at 110°C for 48 h to determine dry weight. Brain water content was calculated as (wet weight − dry weight)/wet weight × 100%.

### Neurological severity score

Neurological dysfunction was evaluated on day 14 post-TBI using the neurological severity score (NSS) according to the protocol of Chen [19]. One point was awarded if the mouse could not finish one of ten tasks. Therefore, maximum score of 10 points indicated severe neurological dysfunction, whereas 0 points represented normal function. All tests were performed by two observers who were blinded to experimental groups and repeated five times to evaluate the average.

### Morris water maze test

The learning ability and spatial memory of mice were assessed using the Morris water maze as previously described [16,20]. An experimental apparatus was divided into four quadrants that was filled with nontoxic white pigments and maintained at 25°C. A round platform was placed 1 cm under the water surface at the midpoint of the fourth quadrant. Each mouse was randomly released in varying quadrants of the apparatus and was allotted 90 s to find the location of the platform that was kept constant. The mice were trained four trials per day for four consecutive days. The test was performed on day 14 post-TBI and four trails were averaged.

### Rotarod test

The motor function of mice was assessed using an automated Rotarod (Ugo Basile, Comerio, Italy). All mice were pretrained before injury at a constant speed of 40 rpm and were tested on day 14 post-TBI. The average latency to fall from the rod was recorded, and the maximum cutoff time was 180 s.

### String test

The string test apparatus consisted of a string (diameter: 2 mm; length: 50 cm) mounted on two vertical supports at a height of 37 cm. Mice were placed on the string midway between the supports and were rated according to the following system: 0 = falls off; 1 = hangs onto the string with two forepaws; 2 = hangs onto the string with two forepaws but attempts to climb onto the string; 3 = hangs onto the string with one hind paw plus two forepaws; 4 = hangs onto the string with two hind paws plus two forepaws; 5 = escape. The string test was performed on day 14 post-TBI and repeated three times.

### Statistical analysis

All data were present as mean ± SEM. *n* value represented the number of independent experiments. The correlation between Ftmt expression and oxidative stress levels was determined by the Pearson correlation test. The behavioral data were analyzed by Kruskal–Wallis test. Comparisons between two groups were analyzed using Student’s *t*-test. All other comparisons were performed by one-way ANOVA with *post hoc* Tukey’s test when it was >2 groups. *P*<0.05 was considered to be statistically significant.

## Results

### TBI decreased Ftmt expression and induced oxidative stress

To evaluate the role of Ftmt in TBI, the expression of Ftmt in injured brain cortex was examined. The Western blotting results showed that Ftmt protein expression was gradually decreased from day 3 to 14 after TBI surgery as compared with sham mice (Figure 1A and B). These data indicate the potential involvement of Ftmt in the TBI-induced brain injuries. Moreover, we also detected the oxidative stress in brain after TBI surgery. The levels of GSH, SOD, MDA, and NO on days 1, 3, 7, and 14 post-TBI were measured. The results showed that brain GSH and SOD levels were gradually decreased after TBI surgery, whereas the MDA and NO levels were gradually increased (Figure 1C and F). The above results suggest TBI is able to induce oxidative stress.

**Figure 1:** TBI decreased Ftmt protein expression and induced oxidative stress in brain cortex (**A**) Ftmt protein expression in mice cortex around injury site on days 1, 3, 7, and 14 post-TBI was determined by Western blotting. (**B**) Quantitative analysis of Ftmt expression after normalization against GAPDH. (**C**–**F**) The levels of oxidative stress indicators GSH (C), SOD (D), MDA (E), and NO (F) in brain were determined by commercial kit as mentioned in method section. Data were present as mean ± SEM; *P<0.05, **P<0.01 versus sham, *n* = 6/group.

### Correlation between Ftmt expression and oxidative stress

We analyzed the possible correlation between Ftmt expression and brain oxidative stress on days 1, 3, 7, and 14 post-TBI using Pearson correlation test. The results showed that the decreased Ftmt expression was positively correlated with GSH and SOD levels with the correlation coefficients (*R*^2^) of 0.6401 and 0.5409 respectively (Figure 2A and B). In addition, Ftmt expression was negatively correlated with MDA and NO levels. The correlation coefficients (*R*^2^) were 0.6815 for MDA level and 0.7897 for NO level (Figure 2C and D). It suggests that the decreased expression of Ftmt may participate in TBI-induced oxidative stress.

**Figure 2:** Correlation analysis of Ftmt expression and oxidative stress by using Pearson correlation test (**A**–**D**) Ftmt protein expression on days 1, 3, 7, and 14 post-TBI was compared with brain levels of GSH (A), SOD (B), MDA (C), and NO (D). The correlation coefficients (*R*^2^) were shown respectively; *n* = 36 mice from six groups.

### Ftmt deficiency enhanced TBI-induced brain oxidative stress

To further explore the effect of Ftmt on TBI-induced oxidative stress, wild-type mice and Ftmt knockout mice were processed for TBI surgery, and the levels of GSH, SOD, MDA, and NO in the brains were assessed respectively. The wild-type and Ftmt knockout mice did not reveal an evident phenotype, including body weight, food consumption, and fertility (data not shown). There were also no significant differences in the levels of GSH, SOD, MDA, and NO between sham wild-type and Ftmt knockout mice. On day 14 post-TBI, the decrease in GSH and SOD levels was more pronounced in Ftmt knockout mice than in wild-type mice. Administration of NAC, a commonly used antioxidant, markedly inhibited TBI-induced the decrease in GSH and SOD levels in wild-type mice. Moreover, NAC dramatically restored the decrease in GSH and SOD levels in Ftmt knockout mice, similar to those observed in NAC-treated wild-type TBI mice (Figure 3A and B). Furthermore, the levels of MDA and NO in Ftmt knockout TBI mice were significantly higher than those in wild-type mice; in contrast, there was no observed increase in NAC-treated Ftmt knockout TBI mice (Figure 3C and D). These results indicate that the TBI-induced oxidative stress could be exacerbated by Ftmt deletion.

**Figure 3:** Effects of Ftmt deletion on TBI-induced brain oxidative stress (**A**–**D**) On day 14 post-TBI, brain cortex extracts from wild-type (WT) and Ftmt knockout (KO) mice with or without N-acetylcysteine (NAC) treatment were analyzed for the levels of GSH (A), SOD (B), MDA (C), and NO (D). Data were presented as mean ± SEM; **P<0.01 versus WT sham; ^##^*P*<0.01 versus WT TBI; ^&&^*P*<0.01 versus KO sham; ^$$^*P*<0.01 versus KO TBI, *n* = 6/group.

### Ftmt knockout exacerbated brain injuries

Oxidative stress has been strongly implicated in the pathophysiology of various brain injuries [7,9]. Given the importance of Ftmt in regulating oxidative stress, we investigated the effect of Ftmt on intracerebral hemorrhage and lesion size induced by TBI. Immunohistochemical staining of mouse IgG revealed that the IgG extravasation in wild-type mice was increased on days 1 and 3 post-TBI as compared with sham mice, indicating the structural integrity of blood–brain barrier is impaired. Compared with WT mice, Ftmt knockout mice showed significantly prolonged hemorrhage in the lesions. However, NAC treatment completely abolished the differences between wild-type and knockout mice (Figure 4A and B). Moreover, the brain infarct volume was determined by TTC staining. As shown in Figure 4C, there was no detectable infarct in sham wild-type and Ftmt knockout mice, while extensive infarction was detected on day 14 post-TBI. Deletion of Ftmt further increased the infarct volume as compared with wild-type mice. Administration with NAC significantly attenuated the enhanced effect of Ftmt knockout on infarct volume, which was similar to those observed in NAC-treated wild-type TBI mice. Additionally, on day 14 post-TBI, brain water content in wild-type and Ftmt knockout mice was both increased as compared with corresponding sham mice, but the increase extent was more noticeable in Ftmt knockout mice. Expectedly, NAC administration also greatly decreased brain edema induced by Ftmt deletion (Figure 4D). These data indicate that Ftmt deficiency further enhances TBI-induced brain injuries.

**Figure 4:** Ftmt ablation aggravated TBI-induced brain injuries (**A**) The brain slides from wild-type (WT) and Ftmt knockout (KO) mice on days 1, 3, and 7 post-TBI were immunohistochemically stained for IgG. (**B**) Quantification of mouse IgG staining intensity; *n* = 6/group, **P<0.01 versus WT. (**C**) The brain infarction was determined by TTC staining and quantitative analysis of the total infarct volume on day 14 post-TBI; *n* = 4/group. (**D**) Brain water content was measured on day 14 post-TBI; *n* = 10/group, **P<0.01 versus WT sham; ^#^*P*<0.05, ^##^*P*<0.01 versus WT TBI; ^&&^*P*<0.01 versus KO sham; ^$$^*P*<0.01 versus KO TBI.

### Ftmt ablation aggravated TBI-induced neurological deficits

Next, we examined whether Ftmt affects neurobehavioral outcomes. For NSS examination, no significant differences could be observed between sham wild-type and Ftmt knockout mice. On day 14 post-TBI, the NSS of wild-type and Ftmt knockout mice was markedly increased as compared with their respective sham mice. Notably, TBI-induced the NSS was higher in Ftmt knockout mice than in wild-type mice (Figure 5A). Furthermore, Morris water maze test showed that sham Ftmt knockout mice took almost the same time to reach the platform as compared with wild-type mice. After TBI surgery, both wild-type mice and Ftmt knockout mice took significantly longer time to reach the platform. However, TBI-treated Ftmt knockout mice exhibited greater memory impairment than TBI-treated wild-type mice (Figure 5B). For motor function analysis, we performed rotarod test and string test. On day 14 post-TBI, wild-type mice and Ftmt knockout mice showed significantly poorer performance on these tasks as compared with their respective sham mice. Furthermore, TBI-induced impairment of motor function was more pronounced in Ftmt knockout mice than in wild-type mice (Figure 5C and D). Inhibition of oxidative stress by NAC ameliorated the above neurological deficits that aggravated by Ftmt ablation (Figure 5A–D). These data suggest that the increased oxidative stress underlies the mechanism by which Ftmt deficiency exacerbates TBI-induced neurological deficits.

**Figure 5:** Ftmt deficiency exacerbated TBI-induced neurological dysfunction (**A**) On day 14 post-TBI, TBI severity was examined by analyzing the neurological severity score (NSS). (**B**) The learning ability and spatial memory of mice were examined by Morris water maze test. The analysis of the recorded data showed the latency to locate the hidden platform. (**C** and **D**) The motor function of mice was assessed by rotarod test (C) and string test (D). The duration on the rotarod and string grip scores was recorded. All data were present as mean ± SEM. **P<0.01 versus WT sham; ^##^*P*<0.01 versus WT TBI; ^&&^*P*<0.01 versus KO sham; ^$$^*P*<0.01 versus KO TBI, *n* = 15/group.

## Discussion

Currently, almost one half of hospitalized patients with severe TBI have irreversible neurocognitive sequelae that significantly influence life quality [2,7]. Unfortunately, although many clinical TBI trials and tremendous progresses have been made in the past decades, the therapeutic options remain limited, such as optimizing cerebral perfusion, treating intracranial hypertension, and providing supportive care, which fail to show a therapeutic benefit, and some even worsen the outcomes [5,16]. Therefore, it is of importance to develop novel strategies for TBI treatment.

Ferritin has been documented to play a key role in the development of various neurodegenerative disorders. A positive correlation between serum ferritin level and peri-hematoma edema volume has been found in patients with spontaneous intracerebral hemorrhage [21]. Recently, Simon and colleagues demonstrated that increased plasma ferritin level correlated with lower Glasgow coma scale scores and predicted fatal outcome following severe TBI [22]. Ftmt, an identified H-ferritin-like protein located in mitochondria, has been reported to be involved in the pathogenesis of Parkinson’s disease, Alzheimer’s disease (AD), and Friedreich’s ataxia [14,20,23,24]. Previous studies have observed increased Ftmt expression in the brains of AD patients, which may play a neuroprotective role against oxidative stress [23,25]. In the present study, we demonstrated that Ftmt expression was gradually decreased after TBI surgery. Moreover, along with the progressive brain injury, the cortex oxidative stress was also increased, as evidenced by reduced GSH and SOD levels and elevated MDA and NO levels. Interestingly, the extent of reduced Ftmt expression in the brain was linearly correlated with oxidative stress on days 1, 3, 7, and 14 post-TBI. Although the correlation coefficients (*R*^2^) were not ideal due to relatively low sample quantity, they were considered to be statistically significant. These above results demonstrate the potential involvement of Ftmt in the oxidative stress following TBI surgery.

Several studies have expanded Ftmt’s therapeutic application by demonstrating that Ftmt can exert a neuroprotective effect against 6-hydroxydopamine- or β-amyloid-induced neurotoxicity [20,26]. On the contrary, β-amyloid-induced neurotoxicity was further exacerbates in Ftmt knockout mice [18]. Inhibition of Ftmt resulted in severe neurodegeneration in the Purkinje cells of the cerebellum [20]. Although the role of Ftmt has been described in multiple neurodegenerative diseases, the neuroprotective effect of Ftmt and its influence on the outcome of TBI remained unclear. There are evidence indicating that oxidative stress is associated with the pathogenesis of TBI [6–8]. Considering the correlation between Ftmt and oxidative stress levels, we initially determined the effects of Ftmt knockout on TBI-induced oxidative stress. In the present study, no significant differences in oxidative stress levels between sham wild-type and Ftmt knockout mice were observed. However, upon TBI insult, the oxidative stress level in Ftmt knockout mice was more pronounced than in wild-type mice, which agreed with a recent study in an AD mice model [18].

Moreover, intracerebral hemorrhage, brain infarction, and edema are the most critical pathological changes of TBI, which are the potential fatal factors leading to death patients [27]. To confirm whether the enhanced effects of Ftmt ablation on oxidative stress could further increase brain injuries, intracerebral hemorrhage, brain infarction, and edema were examined. Our results showed that knockout of Ftmt significantly prolonged hemorrhage in the lesions, suggesting Ftmt down-regulation inhibits the recovery from blood–brain barrier breakdown. Furthermore, Ftmt deficiency also further increased brain infarction and edema. Previous studies have reported that Ftmt deficiency has not any evident phenotype under normal physiological conditions [18,28]. Consistent with these studies, here, we also found that Ftmt knockout mice showed no abnormal behavioral outcomes compared with wild-type mice. However, Ftmt ablation significantly exacerbated TBI-induced memory impairment and dyskinesia, because of their higher NSS and poor performance in the Morris water maze test, rotarod test, and string test. These findings suggest that Ftmt is not necessary under normal conditions, but it appears to exert neuroprotective role after challenge such TBI.

NAC, a well-known antioxidant, is considered by World Health Organization, which may be an important medication need in clinical [29]. The antiapoptotic, anti-inflammatory, and proneurogenic effects of NAC have been described for almost two decades. Moreover, the neuroprotective property of NAC has been reported [30]. Here, with NAC administration, both oxidative stress and neurological deficits in wild-type TBI mice were dramatically attenuated, which consistent with previous study [10,17]. In addition, NAC also inhibited oxidative stress and improved behavioral function in Ftmt knockout mice, similar to the levels of those observed in NAC-treated wild-type TBI mice. These results strongly suggest that the Ftmt deficiency exacerbates brain injuries and neurological deficits at least in part through enhancing oxidative stress after TBI.

In conclusion, the present study reveals that lack of Ftmt exacerbates TBI-induced brain injuries, spatial memory, and neurological deficits through increasing oxidative stress levels. Our findings present a protective role of Ftmt against TBI, suggesting that restoration of Ftmt expression may be a novel therapeutic strategy for the treatment of TBI.

## Abbreviations

Ftmt: ferritin
HRP: horseradish peroxidase
IRE: iron-responsive element
MDA: malondialdehyde
NAC: N-acetylcysteine
NO: nitric oxide
NSS: neurological severity score
OD: optical density
ROS: reactive oxygen species
SOD: superoxide dismutase
TBI: traumatic brain injury
TTC: 2,3,5-triphenyltetrazolium chloride
